# Effects of Acupuncture Combined with Exercise on Expression of Immune Factors in Aging Rats and Its Significance in Antiaging Intervention

This article has been retracted.

**DOI:** 10.1155/2022/6833196

**Published:** 2022-08-16

**Authors:** Lulu Jiang, Hongying Jing, Lan Lan, Xia Liu, Su Wang, Yan Xu, Nijia Meng

**Affiliations:** ^1^College of Sports and Human Sciences, Harbin Sport University, Harbin, China 150008; ^2^College of Sport Humanistic Sociology, Harbin Sport University, Harbin, China 150008

## Abstract

**Background:**

With the improvement of people's living standards, how to maintain health and delay aging to improve the quality of life and achieve longevity has become a hot topic of concern. *objective*. To investigate the effect of acupuncture combined with exercise on the expression of immune factors in aging rats and its significance in antiaging intervention.

**Materials and Methods:**

Forty-three SD rats included 12 rats in the control group, and the remaining rats were injected intraperitoneally with D-galactose 500 mg/kg to prepare a subacute aging rat model. The 24 rats that were successfully modeled were divided into acupuncture exercise groups and exercise groups according to the random number table method, with 12 rats in each group. After the modeling, the comparison group did not do any intervention, the exercise group was given aerobic exercise intervention, and the acupuncture exercise group was given acupuncture combined with exercise intervention. The effect of immune factor expression in rats was compared.

**Results:**

The levels of IgM, IgA, and IgG in the acupuncture exercise group were significantly higher than those in the exercise group (*P* < 0.05). The IL-10 content in the acupuncture exercise group was significantly higher than that in the exercise group (*P* < 0.05) and was significantly reduced in the acupuncture exercise group compared with the comparison group (*P* < 0.05). The level of IL-6 in the acupuncture exercise group was significantly lower than that in the exercise group, and the level of IL-6 in the acupuncture exercise group was significantly increased compared with the comparison group (*P* < 0.05). The C3 and C4 levels in the acupuncture exercise group were significantly higher than those in the exercise group (*P* < 0.05). The levels of IFN-*γ* and TNP-*α* were significantly lower in the acupuncture exercise group than in the exercise group and significantly increased in the acupuncture exercise group compared with the comparison group (*P* < 0.05).

**Conclusion:**

Ling turtle eight method acupuncture combined with exercise promoted the development of immune organ spleen, enhances the body's immune function and complement system, inhibits the immune inflammatory response and regulates immune balance, reduces the inflammatory response caused by the aging of D-type galactose, and achieves the effect of delaying aging.

## 1. Introduction

As our country enters an aging society, aging and related diseases have become increasingly serious social and medical problems [1]. Aging is the decline of the body's immune function from the molecular level, the cellular level, and the organ function level, or even the entire body's immune function, which is a complex physiological and pathological change process and will have a great impact on the body's immune system [2]. With the increase of age, the body's immune system function continues to decline, the body gradually appears a series of degenerative changes, and the prevalence and mortality rate increase significantly [3].

Imbalances in immune function caused by aging can lead to frequent and more severe immune-related diseases [4]. As the immunity of the elderly decreases, the elderly are susceptible to infectious diseases, and the level of response to vaccines is reduced, which in turn increases mortality [5]. Therefore, studying the mechanism of aging to develop drugs and methods to delay aging, enhance the body's ability to resist diseases, improve the quality of health of elderly individuals, and prevent the occurrence of diseases is not only beneficial to individuals but also to the harmony and stability of the whole society and sustainable development [6, 7]. The free radical theory of aging believes that the body's free radical production increases, the level of oxidative stress increases, and the antioxidant function decreases are the main factors leading to aging and shortening life [8]. Exercise is essential for the elderly to stay healthy, which may have antiaging effects. Lack of physical activity causes a variety of skills in the human body, which is manifested at the level of molecules, cells, tissues, organs, and systems. For example, long-term bed rest causes various physiological changes similar to aging and promotes aging. Physical exercise and aerobic exercise are the preferred exercise intensity. Long-term aerobic exercise training can improve people's heart and lung function and enhance people's ability to work aerobically, which has a certain positive effect on delaying aging [9]. Many experiments at home and abroad have proved that appropriate aerobic exercise can enhance the antioxidant capacity of the organism, delay brain aging, and promote learning and memory ability [10]. However, most experiments tend to explore the effect of an aerobic exercise intervention on a single stage of the aging process, and no acupuncture combined with aerobic exercise has been studied [11].

There are many similarities between the understanding and elaboration of aging in Chinese and Western medicines. The application of Chinese health care methods and the concept of treating untreated diseases to delay immune aging-related diseases in Western medicine can be expected to be quite effective [12], and we are particularly interested in the point that if acupuncture combined with aerobic exercise can delay aging, it may also improve the aging organism's ability to respond to vaccines. If acupuncture combined with aerobic exercise can improve the body's ability to respond to vaccines, then whether acupuncture can again be used as a new type of vaccine adjuvant and its introduction into the field of vaccine research will open up another new direction for the combination of Chinese and Western medicines. It will also further promote the study of the mechanism of the effect of acupuncture combined with aerobic exercise.

## 2. Material and Methods

### 2.1. Research Object

Forty-three SD rats included 12 rats in the control group, and the remaining rats were injected intraperitoneally with D-galactose 500 mg/kg to prepare a subacute aging rat model. 24 rats that were successfully modeled were divided into acupuncture exercise group and exercise group according to the random number table method, with 12 rats in each group. Before the experiment, the rats were firstly acclimatized for 1 week, and the laboratory required 12 h of light and 12 h of darkness each day (the light time was 6 : 00~18 : 00), and the room temperature was 19°C~23°C, during which the rats were given water and free food. The “3R” principle was strictly followed throughout the experiment, and the animals were treated following the “Guideline on the good treatment of laboratory animals” issued by the Ministry of Science and Technology of China in 2006 [13].

### 2.2. Aging Rat Model

The senescence model was manufactured using Qin's modeling method [14], in which D-galactose was prepared into 10% D-galactose solution at 500 mg/kg-d with 0.9% saline. The model and intervention group rats were injected intraperitoneally with D-galactose solution once/d daily for 60 d. After 60 d of continuous modeling, the rats gradually showed signs of aging such as yellowing hair, easy hair loss, slow movement, fear of cold, cold extremities, mental depression, and increased urination.

### 2.3. Methods

At the end of the modeling period, the comparison group did not do any intervention, and the aging rats in the exercise group were given aerobic exercise intervention, and the rats swam in a transparent glass tank (160 cm × 60 cm × 110 cm) with a water depth of 80 cm and a water temperature of 34-2°C. After 6 weeks of D-galactose injection, swimming exercise was performed daily at 19 : 00 for 60 min/d for 6 d per week for 4 weeks.

The acupuncture exercise group implemented acupuncture combined with an exercise intervention, the aerobic exercise intervention was kept the same as the exercise group intervention, and the acupuncture intervention was as follows: opening method: according to Xie's simple Ling turtle eight methods for opening acupuncture points, the hour of the day of treatment was selected for opening acupuncture points. The acupuncture points were located according to the “Development of acupuncture point atlas for rats” [15]. The body hair of the acupuncture points was first cut off. A small amount of paraffin oil was applied to the surface of the acupuncture points to fix the moxa cones, and moxibustion was performed without scarring until the rats struggled all over the body, 3 strokes each time, 1 time, for 4 weeks. See Figure 1.

### 2.4. Assay Method

At the end of the experiment, the rats in each group were blooded and executed, and the spleen tissues were quickly taken on an ice table. The spleen tissues were weighed, and 10% spleen homogenate was made with a manual homogenizer. Another 200 mg of spleen tissue was taken and immersed in RNA preservation solution and the activities of serum immunoglobulin M (IgM), immunoglobulin A (IgA), immunoglobulin G (IgG), spleen tissue complement C3, complement C4, interleukin-6 (IL-6), interleukin-10 (IL-10), interferon-*γ* (IFN-*γ*), and tumor necrosis factor-*α* (TNP-*α*) activity.

### 2.5. Observation Indicators

Measurement of spleen index: the spleen tissues were quickly taken from each group of rats on an ice table after execution, washed with physiological saline, blotted on filter paper, and weighed on an electronic balance with an accuracy of 0.001 g, and then, the spleen index was calculated according to the formula: spleen index (mg/g) = (weight of spleen (mg)/weight of rat (g)∗10. Immunoglobulin M (IgM) determination: blood was collected from the ventral vein of each group of rats at the end of the experiment, and the serum was separated by centrifugation at 3000 r/min for 15 min with an ultra-low-temperature centrifuge after blood collection, and the serum was determined by enzyme-linked immunosorbent assay using competitive inhibitory enzyme immunoassay technique. Immunoglobulin A (IgA) and immunoglobulin G (IgG) assay: blood was collected from the vena cava the day after the experiment, and the serum was separated by centrifugation at 3000 r/min in an ultra-low-temperature centrifuge for 15 min after blood collection, and the enzyme-linked immunosorbent assay was used to determine the serum by competitive inhibitory enzyme immunoassay technique. Determination of complement C3 and complement C4 (C3 and C4): rats in each group were executed after blood sampling, and spleen tissues were quickly taken on an ice table, and the spleen tissues were weighed and made into 10% spleen homogenate with a manual homogenizer. The enzyme-linked immunosorbent assay was selected to determine spleen homogenate by competitive inhibition enzyme immunoassay technique, and the operation was largely the same as that of IgM assay. Interleukin-10 and interleukin-6 (IL-10 and IL-6) assay: rats in each group were blooded and executed, spleen tissues were quickly taken on an ice table, spleen tissues were weighed, and 10% spleen homogenates were made with a manual homogenizer. The enzyme-linked immunosorbent assay was selected to determine spleen homogenate by competitive inhibition enzyme immunoassay technique, and the operation was largely the same as that of the IgM assay. Interferon-*γ* (IFN-*γ*) and tumor necrosis factor-*α* (TNF-*α*) assay: the rats in each group were executed after blood sampling, and the spleen tissues were quickly taken on an ice table. The enzyme-linked immunosorbent assay was selected to determine spleen homogenate by competitive enzyme inhibition immunoassay technique, and the operation was largely the same as that of IgM assay.

### 2.6. Statistical Analysis

All statistical data in this study were entered into excel software by the first author and the corresponding author, respectively. The included data were tested by the Shapiro-Wilk method. The mean ± standard deviation (mean±SD) described the measurement data conforming to the normal distribution. The independent sample or paired sample *t*-test was performed within the group, the count data were described by integer or percentage (%), and the *χ*^2^ test was used between or within the group. The included data that did not conform to the normal distribution were described by M(QR), and the Mann-Whitney test was used, and the test level was *α* = 0.05.

## 3. Results

### 3.1. General Information Comparison

Before the experiment, there was no significant difference in the mean age, gender, and weight of the three groups (*P* > 0.05). After the experiment, the spleen index in the acupuncture exercise group was significantly higher than that in the exercise group. The difference was statistically significant (*P* < 0.05) when comparing the acupuncture exercise group with the comparison group. See Figure 2.

### 3.2. Comparison of Serum Immune Indexes

The levels of IgM, IgA, and IgG in the acupuncture exercise group were significantly higher than those in the exercise group, and the differences were statistically significant (*P* < 0.05) in the acupuncture exercise group compared with the comparison group. The IL-10 content in the acupuncture exercise group was significantly higher than that in the exercise group (*P* < 0.05) and was significantly reduced in the acupuncture exercise group compared with the comparison group, and the difference was statistically significant (*P* < 0.05). The IL-6 content in the acupuncture exercise group was significantly lower than that in the exercise group, and the difference was statistically significant (*P* < 0.05) in the acupuncture exercise group compared with the comparison group. See Figure 3.

### 3.3. Immunological Analysis of Spleen Tissue

The C3 and C4 levels in the acupuncture exercise group were significantly higher than those in the exercise group and were significantly reduced in the acupuncture exercise group compared with the comparison group, with statistically significant differences (*P* < 0.05). The levels of IFN-*γ* and TNP-*α* were significantly lower in the acupuncture exercise group than in the exercise group and significantly increased in the acupuncture exercise group compared with the comparison group, with statistically significant differences (*P* < 0.05). See Figure 4.

## 4. Discussion

The decline in the intrinsic physiological functions associated with the organism's aging is responsible for the organism's aging [16]. Conversely, loss of cellular function over time is responsible for cellular senescence, which is cleared by other cells or self-regulates [17]. Senescence occurs in essentially all types of cells during their survival, with different types of cells exhibiting different manifestations of senescence [18]. Immunosenescence is a complex process that is often accompanied by changes in immune-related indicators, thymus, and spleen, which are important immune organs [19]. They play an important role in the differentiation and development of T lymphocytes and B lymphocytes, humoral immunity, and cellular immunity. In addition, thymus index and spleen index are also commonly used to evaluate the immune function of the body [20]. Immunoglobulins are commonly used to evaluate the humoral immune situation. The amount of their content roughly reflects the ability of the body's immune response and the level of humoral immunity of the body. Common changes in immune aging can also be seen in the decrease in the number and functional decline of T and B cells [21]. D-Galactose is a physiological nutrient involved in the metabolism of glucose, but excessive intake of D-galactose will lead to accumulation in the body and conversion of intracellular aldose reductase into galactitol that cannot be metabolized normally [22]. The accumulation of these nonnormally metabolized galactitols in the body will further affect the osmotic pressure of cells, resulting in swelling of cells, increased levels of reactive oxygen species in the body, and damage to cellular biofilm lipids, metabolic disorders, and dysfunction of cells leading to aging [23]. The construction of subacute aging molds using D-galactose has been widely used in experimental studies in China.

In our study, the spleen index of the acupuncture exercise group was significantly higher than that of the exercise group, and the difference was statistically significant, indicating that the Ling turtle eight methods effectively increased the spleen index of the aging model rats, promoted the development of the immune organ spleen and enhanced the immunity of the organism, and effectively delayed aging. This may be due to the fact that the spleen is the largest immune organ in the body, which is the main site of the immune response [24]. The spleen accounts for about a quarter of the total lymphoid tissue in the body, and it contains many T lymphocytes, B lymphocytes, and macrophages, which are important sites of the immune response [25]. In addition, the spleen synthesizes and secures cytokines and complements. It is also an important base for the production of many immune effector factors in the human body, making it an important immune organ in the human body [26]. Spleen quality is positively correlated with immune function. The spleen index reflects the development and immune function of the spleen [27]. Modern studies have shown that the spleen index is significantly higher, and various behavioral indicators in the organism are regulated. Ling turtle eight methods are one of the important components of time acupuncture, which is a perfect combination of meridian theory and Jiu Gong Ba Gua theory [28]. It is to regulate the balance of yin and yang in the human body by using the subtle changes of natural space time in heaven and earth and the law of synergistic changes in the characteristics of the human biological clock, so the combined regulating effect of both meridians and space time regulates the balance of qi and blood in the human meridians and also realizes the holistic view of healing of heaven and man [29].

We have shown that the Ling turtle eight methods effectively increases the content of IgA, IgM, and IgG immunoglobulins in the aging model rats, enhancing the immune function of the body and effectively protecting the body's immune system thus delaying the aging process [30]. IgM is an antibody that appears during the initial immune response and plays an important role in the early response of immune defense. IgM is therefore used to diagnose the presence of infection in the early stages of the disease [31]. IgG is one of the body's most abundant immunoglobulins and is considered the main antibody in the immune response because it has been found to be mainly present in the B-cell immune response [32]. In addition, IgG helps phagocytes improve their ability to phagocytose pathogens and has a good complement activation function. It is able to neutralize free exotoxins and viruses, effectively regulates the phagocytosis of phagocytes, and effectively protects the body's immune system [33, 34]. The presence of large amounts of IgA in human mucosal surfaces and secretory fluids has been found in experiments, and its role is to resist infections by pathogens from the respiratory, intestinal, and urinary tracts via the mucosal epithelium [35]. In addition, IgA binds to monocytes on the mucosal surface and to Fc receptors on the surface of neutrophils, thus phagocytosing pathogens and achieving a regulatory effect, while IgA prevents pathogens from entering cells when they invade them, preventing them from causing cell damage to play a neutralizing role [36].

We found that Ling turtle eight method effectively increased the content of complement C3 and complement C4, which enhanced the complement system of aging model rats and effectively regulated the body's defense function, thus achieving the purpose of delaying aging. C3 and C4 are the two most representative complements in the complement system. Among them, the highest content in human serum and the complement with the highest proportion in the complement system is C3, which is not only one of the important complement components in the innate immune system but also the main point of connection between the conventional and bypass pathways [37]. When immunoglobulins activate the host immune system, complement components of the immune system undergo enzymatic reactions in a fixed order, thus maintaining the defensive, regulatory functions of the body [38]. Complement is an important component of the humoral backbone of the innate immune system, and through host cell reactions, complement enhances phagocytosis of bacteria and clearance of pathogens from the body, strengthening the antimicrobial capacity of complement antibodies [39]. In addition, in the presence of inflammatory mediators, complement components enhance the activity of coagulation factors. In recent years, with the increasing understanding of complement, the scope of complement assay studies has been gradually broadened, complement assay systems have been gradually improved, and more attention has been paid to understand the dynamic changes of complement [40].

We found that Ling turtle eight methods effectively reduced the number of proinflammatory cytokines synthesized at the serum level in rats with the senescence model and attenuated the inflammatory response caused by D-galactose production senescence model to achieve the effect of delaying aging. IL-6 binds to specific receptors on the surface of target cells and activates downstream JAK/STATs and Ras [41]. The biological effects of IL-6 are diverse, and it plays an important role in immune regulation, hematopoietic regulation, and inflammatory response. In the immune system [42], it has been suggested that IL-6 is a proinflammatory cytokine among cytokines, and it has been experimentally demonstrated that there are different degrees of elevated IL-6 levels in conditions such as infection and inflammation, and the level of IL-6 can be used as an indicator of disease severity [43]. After mononuclear macrophages produce IL-6, it participates in the local inflammatory response and inflammatory damage process of the body, promotes cell differentiation, and stimulates cell growth. In the inflammatory response, IL-6 behaves as maintenance of regulatory and effector T cells and inhibits the regulation of CD4+ T cells, while it regulates the expression of endothelial molecules, promotes neutrophil adhesion to vascular endothelial cells towards inflammation, inhibits the regulation of leukocytes, and grows their lifespan. TNP-*α* is a type of proinflammatory cytokine, synthesized mainly by macrophages and monocytes, and TF-*α* in the early TNF-*α* induces the synthesis of monocytes, macrophages, and vascular endothelial cells, which in turn induces the production of multiple proinflammatory factors, increases the overreaction of inflammation, and initiates the inflammatory cascade response, leading to tissue cell infiltration and inflammatory damage through its chemotactic effect on neutrophils, thus causing some damage to the organism [44]. In general, the onset and progression of the disease toward severe disease or the disease has entered the severe stage which can be responded to by the overexpression of TNF-*α*. IFN-*γ* is a type of proinflammatory cytokine that can also be synthesized and secreted by monocytes, macrophages, and other cells and interact with various inflammatory factors [45]. IFN-*γ* can both mediate delayed hypersensitivity responses, enhance the activity of natural killer cells and phagocytosis of macrophages, and increase the uptake of apoptotic cells by macrophages and the synthesis of other inflammatory mediators.

In recent years, many medical practitioners have gradually studied acupuncture to delay aging, both macroscopically and microscopically, with many successes. However, research reports on how to use Ling turtle eight methods to delay aging in temporal acupuncture still need to be explored more deeply. In addition, there are shortcomings in the modeling method of the subacute aging model prepared by D-galactose, and further research on better modeling methods is needed in the future. Finally, the living habits of rats are different from those of humans, and these problems may affect the experiments due to the limitations of experimental conditions. These problems can be the direction and goal of further research in the future. In summary, Ling turtle eight method acupuncture combined with exercise promoted the development of the immune organ spleen, enhanced the body's immune function and the complement system, and effectively regulated the body's defense function while effectively regulating the inflammatory factors in the aging model rats, inhibiting the immune-inflammatory response and regulating the immune balance, reducing the inflammation caused by D-galactose production aging model. The effect of D-galactose on the aging model was reduced, and the effect of delaying aging was achieved.

## Figures and Tables

**Figure 1:** Skeleton and acupuncture points of the rat (1, Shuigou; 2, Baihui; 3, Tianmen; 4, ear tip; 5, Dazhi; 6, Lung Yu; 7, heart front; 8, diaphragm Yu; 9, Jiaozhong; 10, spleen Yu; 11, kidney Yu; 12, Houhui; 13, Huanjiao; 14, Houhai; 15, Yanglingquan; 16, Houshansili; 17, Zhaohai; 18, Sanyinjiao; 19, heel end; 20, Shen pulse; 21, Taichong; 25, knee-front; 26, tail tip; 27, Shenjue; 28, midwrist; 29, front Sanli; 30, Wai guan; 31, nei guan; 32, Quchi; 33, elbow joint; 34, Hegu; 35, finger interval; 36, Houxi; 37, Shenmen; 38, Taiyuan; 39, Shaohai; 40, Shouze; 41, Tanzhong; 42, Chengjiang).

**Figure 2:** General information comparison. The mean ± standard deviation (mean±SD) represents the general information comparison data of our study and the measurement data, and an independent sample *t*-test is performed; the count data is represented by an integer, and the chi-square test is used to find that the three groups of patients before the experiment. There was no significant difference in average age, gender, and weight (*P* > 0.05). After the experiment, the spleen index of the acupuncture exercise group was significantly higher than that of the exercise group, and the acupuncture exercise group was significantly lower than the control group, and the difference was statistically significant (*P* < 0.05).

**Figure 3:** Serum immune index (serum immune index data in our study). The measurement data is expressed by the mean ± standard deviation (mean ± SD), independent sample *t*-test found that the content of IgM, IgA, and IgG in the acupuncture exercise group was significantly higher than that in the exercise group, and the acupuncture exercise group was significantly higher than the exercise group. Compared with the control group, the exercise group decreased significantly, and the difference was statistically significant (*P* < 0.05). The content of IL-10 in the acupuncture exercise group was significantly higher than in the exercise group (*P* < 0.05). The difference was statistically significant (*P* < 0.05). The content of IL-6 in the acupuncture exercise group was significantly lower than that in the exercise group, and the acupuncture exercise group was significantly increased compared with the control group, with a statistically significant difference (*P* < 0.05).

**Figure 4:** Spleen tissue immune analysis (the spleen tissue immune analysis data in our study). The measurement data are expressed as mean ± standard deviation (mean ± SD); independent sample *t*-test found that the content of C3 and C4 in the acupuncture exercise group was significantly higher than that in the exercise group, acupuncture and moxibustion. Compared with the control group, the exercise group decreased significantly, and the difference was statistically significant (*P* < 0.05). The content of IFN-*γ* and TNP-*α* in the acupuncture exercise group was significantly lower than that in the exercise group, and the acupuncture exercise group was significantly increased compared with the control group. There was statistical significance (*P* < 0.05).

## Data Availability

The datasets used and analyzed during the current study are available from the corresponding author upon reasonable request.
